RETRACTED

# MRI Manifestations and Diagnostic Value of Chronic Osteomyelitis

**DOI:** 10.1155/2021/5585676

**Published:** 2021-03-13

**Authors:** Bingyuan Lin, Qiaofeng Guo, Haiyong Ren, Yiyang Liu, Kai Huang

**Affiliations:** ^1^Department of Orthopedics, Tongde Hospital of Zhejiang Province, Hangzhou, Zhejiang 310012, China; ^2^Zhejiang Chinese Medical University, Hangzhou, Zhejiang 310053, China

## Abstract

If chronic osteomyelitis is not treated promptly and thoroughly, the wound will not heal for a long time, and the affected limb will be dysfunctional or disabled. In severe cases, it may even require amputation. In this article, a total of 50 patients with chronic osteomyelitis who meet the inclusion criteria were selected from January 2019 to March 2020 and were divided into two groups based on patient compliance, namely, a treatment group and a control group. The results of this group of studies showed that osteomyelitis is mostly manifested as limited diffusion, showing high signal on DWI, and ADC value is significantly higher than that of normal bone area. The normal bone area did not show obvious focal abnormal signals on the conventional MRI image. The ADC value of the measured patient's osteomyelitis area was compared with the ADC value of the normal bone area. The ADC value was significantly higher than that of the normal bone area, and the difference was statistically significant. Studies have shown that membrane induction technology is superior to the bone handling group in terms of limb function scores and results satisfaction in the treatment of chronic osteomyelitis bone defects. Membrane induction technology has a low complication rate, a small number of X-ray examinations, a short healing time, and a high functional score. However, bone handling technology has a long treatment process, long fixation time and healing time, nail channel infection, joint stiffness, nerve damage, and many other complications.

## 1. Introduction

With the increasing economic development of our country, the number of workers in the industry and construction industry has increased, and rapid transportation such as motor vehicles has become increasingly popular [1]. High-energy injuries caused by machine injuries, fall injuries, and car accident injuries have increased year by year. Such injuries often involve open limb fractures. In addition, due to high-energy damage, it is easy to cause severe trauma to the skin and soft tissues of the fracture, further destroying the blood supply of the fractured end, resulting in difficult fracture healing and the formation of dead bones, thereby providing an adhesion carrier for bacterial growth and bacterial biofilm (BBF) formation. Although the early application of antimicrobial therapy can basically clear the acute bone marrow inflammation after 2–4 weeks, it is difficult to completely remove the local small infectious lesions and bacterial biofilms of the wounded [2]. The local inflammation changes from the acute stage to the chronic course, with repeated attacks and chronic osteomyelitis.

RETRACTED

Chronic osteomyelitis has always been one of the stubborn diseases recognized in the medical profession and is called the “second cancer” [3]. Although the antibacterial activity of the new generation of antibacterial drugs continues to improve, and surgical interventions are becoming more and more perfect, the recurrence rate of chronic osteomyelitis is still as high as 20–30% [4]. Some wounded eventually have to undergo amputation, which not only bring about great physical and psychological pain to the patients, but also impose a heavy economic burden upon the family and the country. It is currently believed that the pathogenesis of chronic osteomyelitis involves a variety of immune and biochemical reactions [5]. Oxidative stress plays an important role in the disease process. It is closely related to the activity of osteoblasts and osteoclasts and wound healing. It is involved in lipid, protein, and genetic damage. The current consensus in the treatment of chronic osteomyelitis is to give antimicrobial treatment on the basis of thorough debridement and wound drainage. Antibacterial drugs run through the treatment of chronic osteomyelitis and determine the success or failure of the treatment. In recent years, despite the continuous introduction of new antibacterial drugs and the continuous improvement of drug delivery methods, the therapeutic effect is not very satisfactory; shortening the treatment time of chronic osteomyelitis, increasing the cure rate, and reducing the disability rate are of great clinical and social significance.

This study analyzed the correlation between ADC value in osteomyelitis area of DF patients and clinical parameters. The results showed that ADC value in osteomyelitis area of DF was negatively correlated with TCPO2 (*r* = −0.498, *P* < 0.05). ADC value in osteomyelitis area and ankle-brachial index (ABI) and toe-brachial index (TBI) have no significant correlation. In this study, ROC curve analysis was performed on the diabetic foot osteomyelitis area and the normal bone area, and the ADC value corresponding to the area under the curve was 0.992, indicating that the ADC value has high sensitivity and specificity, which can be used for clinical diagnosis to provide reliable quantitative imaging parameters. Membrane induction technology surgery is divided into two stages, which has the advantages of fast healing time, fewer complications, and the possibility of its use for emergency surgery. Membrane induction technology can effectively control infection and provide a favorable environment for bone healing. And membrane induction technology has shown obvious advantages in the reconstruction of bone defect after bone tumor surgery. Membrane induction technology and bone transfer technology are two commonly used techniques in clinical treatment of chronic tibial osteomyelitis. This article compares the efficacy of membrane induction technology and bone transfer technology in the treatment of chronic tibial osteomyelitis bone defects and evaluates the two surgical methods.

RETRACTED

The rest of this article is organized as follows.  Section 2 discusses related work.  Section 3 analyzes the pathogenesis and treatment mechanism of chronic osteomyelitis.  Section 4 presents the research objects and methods.  Section 5 discusses the experimental results.  Section 6 summarizes the full text.

## 2. Related Work

The dead bones and nearby scar tissues formed after bone destruction are difficult to achieve due to the lack of blood supply, and the body's own immunity is not enough to fight pathogenic bacteria, so it is difficult to remove drug-resistant strains in the lesion area, which makes the disease prolonged and repeated [6]. Coupled with the general application of antibiotics in the early treatment, the body's immune response and bacterial resistance have basically formed, making the therapeutic effect of traditional antibiotic administration routes such as oral and injection difficult to achieve the expected goal. *Staphylococcus aureus* is the most common pathogen of chronic osteomyelitis [7]. After research, relevant scholars have found that the presence of *Staphylococcus aureus* can be detected in 50%–75% of patients with chronic osteomyelitis [8]. *Staphylococcus aureus* and *Staphylococcus epidermidis* can form a layer of biofilm with polysaccharide–protein complex as the main component on the surface of bone or internal fixation. The bacteria will initially adhere to the surface of the colony, and then the bacteria and bacteria will adsorb each other to form a multilayered bacterial network, and finally the bacteria will reach the resting or dormant period to complete the entire biofilm formation process [9]. Biological organisms rely on the multilayer protection formed by biofilms, which can effectively avoid opsonin, phagocytosis, and antimicrobial agents and resist clinical antibiotic treatment and the elimination of bacteria by phagocytes of the immune system, so as to achieve the purpose of protecting bacteria [10]. In addition, the lack of reasonable use of antibiotics for a period of time further increases the resistance of bacteria. These are important factors that constitute the difficulty of curing chronic osteomyelitis and the high recurrence rate.

RETRACTED

Related scholars proposed the combined use of amoxicillin and gentamicin to eliminate Gram-positive and Gram-negative bacteria, and the efficacy was confirmed through experiments [11]. Local application of antibiotics not only reduces the liver and kidney toxicity and drug resistance caused by systemic antibiotics, but also effectively increases the local inhibitory concentration. For example, the antibiotic polymethyl methacrylate (PMMA) and calcium sulfate release systems are both common antibiotic bone cements in clinical practice. This method can not only control infection by local drug concentration, but also rely on surgical removal of dead bones to fill the defect area with bone cement to achieve the purpose of maintaining limb stability [12]. However, this method also cannot completely control the infection. When the defect area is too large, such as the length of the defect is greater than 10 cm, then the bone cement filling alone cannot maintain the force line of the tibia and bear the body weight, resulting in the patient's long-term bed rest and early joint dysfunction.

Conventional MRI has now become an imaging method for detecting bone and soft tissues involved in osteomyelitis and has certain value for the diagnosis of osteomyelitis [13]. Relevant scholars pointed out that the osteomyelitis signal changes can be found in the early stage of the disease, which are mainly manifested as low signal on T1WI, high signal on T2WI, high signal of fat suppression sequence, and enhanced scanning [14]. Osteomyelitis mostly originates from surrounding soft tissue infection and ulcer formation. The infection invades adjacent bone through damaged skin or broken bone cortex and then causes corresponding bone infection. Because the forefoot and heel are the main weight-bearing parts of the foot, skin ulceration is likely to occur here, which can cause foot soft tissue infections, so osteomyelitis mostly affects the forefoot and heel.

Related scholars have found that the pathogenic bacteria of chronic osteomyelitis can produce polysaccharide-protein complexes [15]. The bacteria adhere to the dead bone to form a biofilm. Under the protection of the biofilm, the bacteria can latent and breed in the dead bone. In order to destroy the bacteria in the biofilm, the concentration of antibiotics must be increased. Chronic osteomyelitis has extremely poor local blood circulation. It is difficult for the whole body to use antibiotics to reach the lesion through the blood circulatory system, and the antibiotics that penetrate into it are far from reaching the effect of killing the bacteria in it. Pathological studies have shown that there will be a patchy fibrous interval between the chronic osteomyelitis lesion and the normal tissue [16]. The blood circulation in the scar fibrous interval is extremely poor, and the blood supply of the corresponding tissue in the lesion is also very poor, even with high blood drug concentration. The amount of drug that can penetrate into the lesion tissue may not be enough to kill the bacteria in it.

RETRACTED

Relevant scholars found 66 strains of pathogenic bacteria in 96 cases of osteomyelitis, of which Gram-positive bacteria accounted for 51.52%, and Gram-negative bacteria were mainly *Pseudomonas aeruginosa* [17]. This shows that chronic osteomyelitis has caused chronic osteomyelitis in recent years. The bacteria have undergone major changes, and the infection rate of Gram-negative bacteria has increased significantly. Vancomycin is a glycopeptide macromolecular antibiotic. It has a strong potency and is often used when other antibiotics are ineffective against bacteria. Vancomycin has an incomparable effect in the treatment of Gram-positive cocci. In recent years, it has been used more and more in the treatment of bone infections [18–20]. It basically treats all pathogens that may cause chronic osteomyelitis.

For chronic osteomyelitis, bone defects often occur during the treatment process, and bone graft repair is needed to promote bone healing. The current repair techniques mainly include autologous or allogeneic bone transplantation, xenogeneic bone transplantation, implantation of artificial bone and biomaterial substitutes, and autologous bone lengthening. At present, most scholars believe that autologous bone transplantation is the gold standard for bone transplantation, because it can provide good osteoconductivity and osteogenesis, and there is no immune rejection reaction; moreover, there is no risk of disease transmission [21–23]. The disadvantage is the autologous bone transplantation suffering. Due to the limitation of material extraction, large amounts of bone cannot be taken, and large bone defects cannot be repaired. Allogeneic bone grafts are often considered contraindicated in the repair of infectious bone defects. However, related scholars used allogeneic bone transplantation to treat 32 cases of bone defects formed after thorough expansion of chronic osteomyelitis [24]. The average follow-up was 28 weeks. 29 cases (91.43%) did not reappear infection and achieved good bone healing. However, due to the rejection reaction of allogeneic bone, its widespread clinical application still needs further verification.

RETRACTED

## 3. Pathogenesis and Treatment Mechanism of Chronic Osteomyelitis

### 3.1. Pathogenesis of Chronic Osteomyelitis

Under normal circumstances, a certain number of pathogenic bacteria can exist in the human body, but only under certain conditions can cause disease. This depends on the relationship between the pathogenic bacteria and the body, mainly including patient resistance. The incidence of acute osteomyelitis mainly depends on the relationship between the body's resistance and the virulence of pathogenic bacteria. The human body's resistance includes systemic resistance and local resistance and has the function of preventing pathogenic bacteria from entering the human body and eliminating pathogenic bacteria. The overwhelming majority of chronic osteomyelitis is caused by delayed or improper treatment of acute osteomyelitis and delayed development of the disease. The onset of the disease can also be subacute or chronic. If the patient's resistance is strong, the pathogenic bacteria of acute osteomyelitis are low in virulence and the number is small; it can be manifested as subacute osteomyelitis or chronic at the beginning of the disease osteomyelitis and no obvious acute symptoms. The diagnosis diagram of chronic osteomyelitis is shown in Figure 1.

Whether it is transformed from acute osteomyelitis or a chronic process at the beginning of the disease, the pathological changes are similar, manifested as bone destruction and sequestered bone formation, with new bone in the later stage, becoming bony cladding. The pathological evolution of acute osteomyelitis is the premise and basis for the development of chronic osteomyelitis. A large number of bacterial thrombi are retained, blocking the small blood vessels supplying bone blood, and osteonecrosis can occur rapidly, accompanied by local congestion, exudation, and leukocyte infiltration. The proteolytic enzyme released by leukocytes destroys bacteria, necrotic bone tissue, and adjacent bone marrow tissue. Exudates, dead white blood cell groups, and destroyed bone fragments become small abscesses and gradually increase, making the hard bone marrow cavity with limited capacity higher pressure, causing other blood vessels to be compressed, and forming more necrotic bone tissue. The clinical manifestation is an increasing focal abscess, and the pus can spread along different routes.

### 3.2. The Reasons Why Chronic Osteomyelitis Is Difficult to Cure and Repeated

The extracellular matrix produces a biofilm on the surface of the bacteria, which can protect it from being cleared by antibiotics and phagocytes. Therefore, even with a high blood drug concentration, the drug that can penetrate into the lesion tissue is minimal. It is impossible to kill the living bacteria in the lesion and penetrate the bacterial biofilm. In addition, the bacteria in the chronic inflammation phase grow slowly and are basically in the static phase, while antibiotics have a greater bactericidal effect on the bacteria in the active phase. Therefore, the existence of dead bones in the lesion, the harsh environment of ischemia and hypoxia, and the special drug resistance of bacteria are considered to be the reasons why chronic osteomyelitis is difficult to cure and easy to relapse. In addition, the patient's “long-term illness must be deficient” has low autoimmune function and low surgical tolerance, and the treatment of chronic osteomyelitis is even more difficult.

RETRACTED

The more commonly used methods for the treatment of chronic osteomyelitis include butterfly surgery, muscle flap packing, closed lavage, PMMA bead chain implantation, and open bone grafting. Although there are many methods and they are different, the treatment principles are basically the same. It is to completely remove the lesion as much as possible, remove the dead bone, remove the hypertrophic scar and granulation tissue, eliminate the dead space, reasonably repair the soft tissue defect, improve the local blood circulation, and actively fight the infection. After the infection is controlled, the bone defect will be repaired and closed. The wound is clinically cured. Due to the long course of chronic osteomyelitis, traditional methods will inevitably encounter many problems in the operation process. For example, antibiotic lavage and drainage treatment of chronic osteomyelitis has the main disadvantages of easy clogging of the tube, poor drainage, and the need for secondary tube placement. Local washing speed is limited, bacteria and necrotic tissue cannot be completely removed, and long-term intubation is easy to cause cross-infection; simple antibiotic bone cement bead chain implantation cannot guarantee the soft tissue conditions around the lesion, and it is a second-stage soft-tissue repair. This causes difficulties, leading to the need for extensive muscle or skin flap transplantation to prolong the course of the disease; open bone grafts need to be combined with the application of long-term systemic antibiotics, which have certain toxic and side effects on important organs of the body, and the body is also prone to drug resistance. Therefore, the clinical treatment of chronic osteomyelitis still has a high recurrence rate. In addition to the above, the reasons for the incurable disease and recurrence may also be related to insufficient drainage time and insufficient antibiotic application.

RETRACTED

### 3.3. Application Mechanism of Negative Pressure Closed Drainage Technology in the Treatment of Chronic Osteomyelitis

There are two main explanations for the underlying mechanisms of the VSD technology in the treatment of chronic osteomyelitis: continuous negative pressure suction and the application of mechanical mechanics. Continuous negative pressure drainage can not only reduce molecular interstitial pressure, reduce the edema of the lesion, shorten the diffusion distance, promote the growth of microvessels, and increase blood supply, but it can also remove the fallen necrotic tissue, exudate, bacteria, and soluble harmful substances. The wound surface of the lesion is covered with dressing, which can promote the formation of granulation tissue under negative pressure mechanical shaping. The technical route of VSD is shown as in Figure 2.

VSD is only a part and a link in the treatment of chronic osteomyelitis. Its biological action principle has not yet been fully elucidated. For the treatment of chronic osteomyelitis, thorough debridement of the lesion site, reasonable application of antibiotics, and soft tissue coverage of the wound site are the key to treatment, and they are also issues that need to be considered before VSD coverage and sealing.

### 3.4. Application Mechanism of Antibiotic Bead Chain Implantation in the Treatment of Chronic Osteomyelitis

Although VSD has many advantages in the treatment of chronic osteomyelitis, it is not the ultimate means to treat chronic osteomyelitis as a physical method. The complete removal of bacteria ultimately requires the action of antibiotics. Due to the extremely poor local blood supply in chronic osteomyelitis, the hardening of the cavity wall left after bone destruction, and the resistance of the biofilm on the bacterial surface, it is difficult for simple intravenous antibiotics to enter the bone cavity; antibiotics are added through lavage, even if the lavage rate does not guarantee sufficient time for antibiotics to exert their bactericidal effects. Therefore, the key step in the treatment of chronic osteomyelitis is how to ensure and maximize the bactericidal effect of antibiotics after debridement and drainage. A large number of clinical data have proved that the local application of implanted antibiotic beads to the lesion can achieve an effective bactericidal concentration at the lesion and avoid the side effects of systemic antibiotics.

After the antibiotic beads are removed for the second time, the appropriate treatment is selected according to the scope of the bone defect. If the bone defect is small in scope, it can be directly grafted with autologous iliac bone; if the scope is larger, it can be treated with the Ilizarov external fixator technique. In order to avoid the damage of the second operation and the reconstruction of the cavity after the beads are removed, it provides osteoconductivity, increases the osteoinductive activity, and promotes the repair of bone defects. However, the structural integrity of biodegradable materials often changes during the degradation process. It is difficult for endoplants to maintain the structural integrity, and the degradation rate is inconsistent with the growth rate of new bone. Its osteoinductive activity cannot meet the needs of bone defects. In addition, there is still a lack of data that can prove the effectiveness of degradable material drug delivery systems. For these reasons, degradable antibiotic beads have not been widely used in clinical practice.

RETRACTED

## 4. Research Objects and Methods

### 4.1. General Information

The research objects in this article originate from patients with chronic osteomyelitis who were hospitalized in Wendeng Osteopathic Hospital from January 2019 to March 2020. Patients are divided into two groups according to their personal compliance. The treatment group included 18 males and 7 females, aged 24 to 46 years, with an average of 33.8 years, and a medical history of 5 to 15 months; in the control group, 20 males and 5 females, aged from 25 to 49 years, with an average of 36.0 years, the medical history is 6–16 months. A total of 50 patients in the treatment group and the control group were hospitalized for complete treatment, and no cases were excluded or missed.

### 4.2. Diagnostic Criteria

According to the third edition of “Practical Orthopedics,” the diagnostic criteria were developed.

① Have a history of open fractures and local soft tissue contusion fractures.

② Sinus formation, discharge of purulent secretions, repeated attacks, long-term nonunion, peripheral pigmentation, inflammatory granulation tissue at the mouth of the sinus, and sometimes small pieces of dead bone can be discharged. It may be accompanied by symptoms such as aversion to cold, fever, local redness, swelling or lumps, pain, and discharge of pus. There may be no systemic symptoms during the quiescent period of inflammation. The affected limb joints may have varying degrees of dysfunction.

③ Local soft tissue defect, exposed bone, redness, pain, and pus.

④ It can be seen that the bone is thickened and hardened, the bone marrow cavity is irregular, and there are dead bones of different sizes. It can be seen that the fracture does not heal and the false joint is formed.

Comply with items ① and ④ above, plus any one of items ② and ③, and exclude bone tumors, bone tuberculosis, syphilitic osteomyelitis, etc., to constitute a diagnosis.

RETRACTED

### 4.3. Exclusion Criteria

The exclusion criteria for chronic osteomyelitis in this article are as follows:

  ① Those who do not meet the above diagnostic criteria for chronic osteomyelitis.
  ② Persons under the age of 20 or over 75.
  ③ Those who cannot adhere to the prescribed medications.
  ④ Severe bone damage and loss of limb function.
  ⑤ Combined with large area bone defect.
  ⑥ Patients with severe cardiovascular, liver, kidney, or hematopoietic system.
  ⑦ Does not meet the inclusion criteria, fails to use the prescribed drugs, and cannot determine the efficacy.
  ⑧ Women who are breastfeeding or are about to become pregnant.
  ⑨ Those with allergies and allergies to multiple drugs.
  ⑩Patients with sepsis; patients who suspend treatment without authorization or fail to complete regular follow-up during hospitalization; and patients who withdraw from treatment by themselves.

### 4.4. Research Methods

Some abnormal indicators are corrected to achieve the conditions suitable for tolerating surgery. According to the patient's main complaint and physical examination, reasonable imaging examinations of the limbs' lesions, including routine X-ray examinations, are carried out. If the X-ray film fails to fully reflect the location of the lesion, an MRI examination should be performed to have an accurate understanding of the specific situation of the lesion, so as to facilitate the development of a surgical plan.

After admission, the sinus condition of the infected lesions was routinely treated by intravenous infusion of broad-spectrum antibiotics, and sinus secretions were taken for bacterial culture and drug sensitivity test. Three days before the operation, according to the results of the susceptibility test of sinus bacterial culture, the corresponding antibiotics were selected, and the treatment was given by intravenous drip. After the operation, under the condition that the patient's body function is stable, patients continue to receive effective antibiotic treatment.

The first stage is debridement and fixation. First, we make a plan before surgery and completely remove the bone scar under direct vision. After the bone tissue and dead space without blood supply are fully exposed, we remove them all. At the same time, the hardened bone surface around the dead bone is cleaned until the wound is debrided until fresh blood leaks out of the surrounding bone surface. When the debridement process comes to an end, we use hydrogen peroxide, physiological saline, and type III Aner iodine to repeatedly wash, soak, and rinse the wound cavity 3 times until the wound is clean. After debridement, there is often instability between the two sections of the lesion, and an external fixator should be used at this time. Then we cover the wound with VSD foam, paste biofilm, connect the negative pressure device, and carefully check for air leakage.

RETRACTED

The second stage is bone grafting. After removing the VSD material, we leave the VSD biofoam for bacterial culture and drug sensitivity. If there is no obvious purulent secretion in the lesion and the growth of fresh granulation tissue can be seen, autologous cancellous bone transplantation is performed in the bone defect area. We use hydrogen peroxide, normal saline, and type III Aner iodine to repeatedly rinse, soak, and rinse the lesion area 3 times. Later, a number of cancellous bones are taken from the iliac bone, made into fine particles, filled in the cavity area of the lesion, and compacted. Finally, we cover the surface of the cancellous bone and the lesion with VSD, stick a film, and turn on the negative pressure for continuous suction.

The third stage is to repair skin and soft tissue defects. After the VSD is removed, if fresh granulation growth and no purulent secretions are visible on the surface of the cancellous bone, blood oozing from the wound is routinely collected and retained for bacterial culture. Afterwards, the lesion was repeatedly washed, soaked, and washed 3 times with hydrogen peroxide, normal saline, and type III Aner iodine. Finally, according to the specific conditions of the skin and soft tissue around the bone graft, the method of closing the wound can be selected, such as skin grafting or vascularized transfer flaps. (Note: Before bone grafting, VSD needs to be replaced every 7–10 days. The number of times to replace VSD is determined according to the amount of purulent secretions and necrotic tissue in the lesion after VSD is removed, until freshness is visible in the lesion. Bone grafting is only possible when granulation tissue is available.)

### 4.5. Statistical Methods

All data were processed by statistics: statistical analysis was performed with SPSS16.0 statistical software. Two independent sample *t*-tests are performed for measurement data comparison, *t* test or rank sum test is performed when variance is not uniform, and chi-square test or Fisher's exact probability method is performed for count data. When *P* < 0.05, the difference is considered statistically significant, when *P* < 0.01, the difference is considered statistically significant, and when *P* > 0.05, the difference is considered not statistically significant.

## 5. Results and Analysis

### 5.1. Routine MRI Findings and Location of DF Osteomyelitis

The MRI manifestations of the 6 cases of chronic osteomyelitis in this article are shown in Figure 3. Osteomyelitis manifests as low signal on conventional T1WI and high signal on T2WI. The enhanced scan is obviously enhanced. Osteomyelitis mostly affected the metatarsals and phalanges. In this study, 6 cases involved the phalanges, 3 cases involved the metatarsals, 5 cases involved the metatarsals and phalanges, and 1 case involved the metatarsals, phalanges, cuneiform bones, and scaphoid bones. Among the signs of osteomyelitis, 8 cases were accompanied by swelling of surrounding soft tissues, 7 cases were accompanied by adjacent skin ulcer formation, 1 case was accompanied by sinus and abscess cavity formation, and 2 cases were accompanied by multiple local bone destruction and absorption.

RETRACTED

### 5.2. ROC Curve Analysis of DF Osteomyelitis Area and Normal Bone Area

The ROC curve analysis of the DF osteomyelitis area and the normal bone area shows that the ADC value is located on the dividing line. When the ADC cut-off value is 1.21 × 10^−3 ^mm^2^/s, the diagnostic sensitivity and specificity are both 91.5%. As shown in Figure 4, the abscissa represents 1−specificity, the ordinate represents sensitivity, and the area under the ADC value curve is 0.76.

### 5.3. Correlation Analysis of ADC Value in DF Osteomyelitis Area and Clinical Parameters ABI, TBI, and Tc PO2

Pearson's correlation analysis showed that ADC value in osteomyelitis area of DF patients was negatively correlated with Tc PO2 (*P* < 0.05), and ADC value in osteomyelitis area was not significantly correlated with ABI and TBI (*P* < 0.395 and *P* < 0.507), as shown in Figure 5.

### 5.4. Comparison of the Treatment Results of the MRI Membrane Induction Group and the Bone Transport Group

The membrane induction technology group was better than the bone removal group in the cure time, MRI frequency, and full-weight-bearing time (*P* < 0.05). There was no significant difference in the follow-up time between the membrane induction technique group and the bone transport technique (*P* > 0.05). The comparison of the treatment results of the two groups of patients is shown in Figure 6.

In this study, the last postoperative knee HSS score, ankle AOFAS score, and Maryland foot score were better than those before surgery, and the difference was statistically significant (*P* < 0.05), indicating that the two surgical methods are both effective in the treatment of chronic osteomyelitis bone defects. The last postoperative knee HSS score, ankle joint AOFAS score, and Maryland foot score were better than those in the bone handling technique group, and the difference was statistically significant (*P* < 0.05). The reason may be that the healing time of the bone handling technique is related to the length of the bone defect. For large-scale bone defects, the external fixation frame is longer, which affects the functional exercise of the affected limb and causes the stiffness of the knee or ankle joint. In this study, the second-stage operation of the media induction technique group used internal fixation, which was well tolerated by patients and could strengthen the functional exercise of the affected limb early and reduce the occurrence of joint stiffness. The membrane induction technology group was better than the bone removal group in the cure time, total hospitalization cost, number of X-rays, and full-weight-bearing time (*P* < 0.05). The advantage of bone handling technology is that it can bear weight immediately after surgery. In addition, bone handling technology can continuously adjust the length of the limbs through external fixation and can perform one-stage surgery on infected bone defects. In the case of soft tissue defects, the limbs can be shortened so that the soft tissue can be covered.

RETRACTED

### 5.5. Comparing the Complications of MRI Membrane Induction Group and Bone Transport Group

In the membrane induction technology group, there were 3 complications, 1 joint stiffness, 1 infection recurrence, and 1 incision infection, and the total incidence of complications was 18.72%. There were 7 complications in the bone handling technology group, 2 cases of nail tract infection, 2 cases of infection recurrence, 2 cases of incision infection, and 1 case of joint stiffness, and the total incidence of complications was 56.1%. The total incidence of complications in the membrane induction technology group was lower than that in the bone handling technology group. After statistical data analysis of the complications of the two groups, the difference in complications between the two groups was statistically significant (*P* < 0.05). The comparison of complications between the two groups is shown in Figure 7.

There were 3 complications in the membrane induction technology group, 1 case of joint stiffness, 1 case of infection recurrence, and 1 case of incision infection. There were 7 complications in the bone handling technique group, 2 cases of nail tract infection, 2 cases of infection recurrence, 1 case of incision infection, and 2 cases of joint stiffness. The total incidence of complications in the membrane induction technique group was lower than that of the bone handling technique group. The complications of the two groups were statistically different (*P* < 0.05). In this study, there was 1 case of infection recurrence in the membrane induction technique group. It was considered that the primary debridement was insufficient and excessive autogenous bone was preserved, resulting in uncontrolled primary surgical infection. After the second debridement, the implantation of bone cement can be controlled. The main complication of the two groups of surgery is infection, so radical debridement is essential in the first stage, especially for infectious bone defects. Osteomyelitis is a kind of biofilm inflammation. Mature bacterial biofilms can resist host immunity and antibiotics. In addition, the internalization of bacteria and the presence of local soft tissue infections will cause the debridement to fail. Incomplete debridement is an important factor for recurrence of infection. Only by completely removing the lesions that preserve the bacterial biofilm, such as implants, dead bones, scars, and granulation, can the risk of infection recurrence be reduced. If intramedullary infection occurs, the hole should be reamed and flushed. The main complications of membrane induction technology are joint stiffness, incision infection, and bone cement allergy. Complications of bone handling technology mainly include joint contractures, disuse atrophy, stress fractures, and complications of nonunion or delayed union of the joints.

RETRACTED

### 5.6. Comparing the Functional Scores of the MRI Membrane Induction Group and the Bone Transport Group

Using two independent sample *t*-tests, the membrane induction technology group was better than the bone removal technology group in the last knee HSS score, ankle AOFAS score, and Maryland foot score in this study, and the difference was statistically significant (*P* < 0.05). The HSS score of the knee joint, AOFAS score of the ankle joint, and the Maryland foot score of the two groups of patients after operation were better than those before the operation, and the difference was statistically significant (*P* < 0.05). There was no significant difference between the two groups of patients in the preoperative knee HSS score, ankle AOFAS score, and Maryland foot score (*P* > 0.05). The knee HSS scores, ankle AOFAS scores, and Maryland foot scores of the two groups of patients are shown in Figures 8–10.

### 5.7. Comparative Analysis of DWI Performance and ADC Value between DF Osteomyelitis Area and Normal Bone Area

Two experienced imaging doctors used GE ADW 4.4 imaging workstation Functool software to measure the apparent diffusion coefficient (ADC). In this study, patients were divided into osteomyelitis areas and normal bone areas based on whether there were abnormal inflammatory signals on conventional MRI images. We selected the upper and lower 4 layers of lesions in the osteomyelitis area as the area of interest. The ROI avoids blood vessels, muscles, necrosis, and cystic area, and the size is set to 20–25 mm^2^. In the normal bone area far from the osteomyelitis area, the upper and lower 4 ROIs were measured, respectively, and the average value of the 4 ROIs was taken as the final measurement result and used for statistical analysis. The ROI was manually drawn by two radiologists who have worked for more than 10 years, and when they disagree, they will be determined after consultation and discussion.

RETRACTED

Normal bone is low signal on DWI, osteomyelitis is high signal on DWI, ADC value of normal bone is about 0.81 ± 0.12 × 10^−3 ^mm^2^/s, ADC value of osteomyelitis is about 1.41 ± 0.11 × 10^−3 ^mm^2^/s, the ADC value of the quantitative parameter in the osteomyelitis area of the patient was significantly higher than that of the normal bone area, and the difference was statistically significant (*P* < 0.05). The MRI appearance of DF osteomyelitis area is shown in Figure 11.

## 6. Conclusion

This article improves the traditional open bone grafting technology by introducing the VSD continuous negative pressure suction technology, fully integrates the advantages of the two, and provides a new treatment idea for the treatment of chronic osteomyelitis. This article compares the clinical efficacy of improved open bone grafting technology and traditional open bone grafting technology in the treatment of chronic osteomyelitis. The purpose is to find a therapeutic method for the treatment of chronic osteomyelitis that is effective, safe, and reliable. The DWI and ADC values of patients with DF osteomyelitis have certain clinical application value in distinguishing the osteomyelitis area from the normal bone area. There was no significant difference in general data between the membrane induction technology group and the bone handling technology group (*P* > 0.05). Membrane induction technology group was better than bone removal technology group in terms of cure time, total hospitalization cost, number of X-rays, and full-weight-bearing time, and the difference was statistically significant (*P* < 0.05). The total incidence of complications in the membrane induction technology group was lower than that in the bone handling technology group, and the difference was statistically significant (*P* < 0.05). The membrane induction technology group was better than the bone handling technology group in the last knee HSS score, ankle AOFAS score, and Maryland foot score in this study, and the difference was statistically significant (*P* < 0.05). The HSS score of the knee joint, AOFAS score of the ankle joint, and the Maryland foot score score of the two groups of patients were better than those before the operation, and the difference was statistically significant (*P* < 0.05). There was no significant difference between the two groups of patients in the preoperative knee HSS score, ankle AOFAS score, and Maryland foot score (*P* > 0.05). However, due to the small amount of this study, longitudinal follow-up of patients with osteomyelitis was not performed to analyze the disease progression and healing of patients with osteomyelitis, and only the difference in ADC values between the osteomyelitis area and the normal bone area was analyzed. With the increasingly mature isolation, culture, induction and expansion techniques, EPCs can be obtained relatively easily from peripheral blood or bone marrow. Through research, it provides experimental and theoretical basis for the clinical use of EPCs to promote vascularization tissue engineering bone conjunctival membrane induction technology to repair large-scale bone defects. If the study proves that the EPCs-promoting vascularization tissue engineering osteoconjunctival membrane induction technology is indeed effective in repairing large bone defects, then this technology has a good application prospect.

RETRACTED

## Figures and Tables

**Figure 1:** Schematic diagram of the diagnosis of chronic osteomyelitis.

**Figure 2:** VSD technical route.

**Figure 3:** MRI findings of 6 cases of chronic osteomyelitis.

**Figure 4:** ROC curve analysis of ADC values in DF osteomyelitis area and normal bone area.

**Figure 5:** Correlation analysis between ADC value and ABI, TBI, and Tc PO2 in osteomyelitis area.

**Figure 6:** Comparison of treatment results between the two groups of patients.

**Figure 7:** Comparison of complications between the two groups.

**Figure 8:** HSS scores of knee joints in the two groups.

**Figure 9:** AOFAS score of ankle joint.

**Figure 10:** Maryland foot score.

**Figure 11:** MRI appearance of DF osteomyelitis area.

## Data Availability

The data used to support the findings of this study are available from the corresponding author upon request.
